# Clinical Observation on the Nursing Effect of Mindfulness-Based Stress Reduction Combined with Solution-Focused Brief Therapy in Uremic Peritoneal Dialysis Patients and Influence on Nutritional Status

**DOI:** 10.1155/2021/3751585

**Published:** 2021-09-24

**Authors:** Yiqian Wang, Huazhi Lin, Lihua Wang, Jun Cao, Dan Zheng, Jing Zhu

**Affiliations:** Department of Nephrology, The First People's Hospital of Wenling, Wenling, Zhejiang 317500, China

## Abstract

**Objective:**

To explore the nursing effect of mindfulness-based stress reduction (MBSR) combined with solution-focused brief therapy (SFBT) in uremic peritoneal dialysis (PD) patients and its influence on nutritional status.

**Methods:**

A prospective study was conducted on 108 uremia patients undergoing PD who were admitted to the First People's Hospital of Wenling from March 2018 to December 2020. In accordance with the wishes of the patients, according to random number method, the patients were divided into control group (*n* = 54) and experimental group (*n* = 54). Patients in the control group were given routine care. Patients in the experimental group were given MBSR combined with SFBT. The clinical data, biochemical indicators, complication, compliance, nutritional status, and quality of life of the two groups were compared.

**Results:**

After intervention, the serum hemoglobin, serum albumin levels, and urea clearance index of the experimental group were higher than those of the control group (*P* < 0.05). Compared with the control group, the experimental group had a lower incidence of complications (*P* < 0.05). After intervention, the compliance score of the experimental group was higher than that of the control group (*P* < 0.05). After intervention, the malnutrition inflammation score of the experimental group was lower than that of the control group (*P* < 0.05). After intervention, the Kidney Disease and Quality of Life-36 scores of the experimental group were higher than those of the control group (*P* < 0.05).

**Conclusion:**

MBSR combined with SFBT has a good nursing effect in uremia patients undergoing PD and can increase the patient's treatment compliance, improve the quality of life, and improve the nutritional status.

## 1. Introduction

Uremia is a common clinical syndrome of various advanced kidney diseases, and it is a syndrome composed of a series of clinical manifestations that appear when chronic kidney failure enters the terminal stage. The main clinical manifestations of uremia are edema, fatigue, loss of appetite, metabolic acidosis, water, and electrolyte balance disorders and other manifestations, which can seriously affect people's quality of life [1, 2]. At present, peritoneal dialysis (PD) has become one of the main clinical treatments for uremia, which can effectively alleviate the symptoms of end-stage renal disease, and is preferred by many patients with uremia [3]. PD is a treatment method that uses the semipermeable membrane properties of the human body's own peritoneum and pours peritoneal dialysate into the abdominal cavity to remove water and toxins. It has a good protective effect on the residual renal function and has the advantages of simple operation, no need to establish vascular access, and no need for special equipment, and the treatment can be completed independently at home [4]. However, in uremia as a chronic disease, in the process of long-term acceptance of PD, there is not only long treatment cycle but also high economic costs. With the progress of treatment, uremia patients undergoing PD will inevitably experience a certain degree of discomfort, which aggravates the physical and psychological burden of patients and further aggravates the complications caused by the disease [5]. At the same time, the uremia patients who received PD had low confidence in maintenance treatment, and the degree of cooperation with medical staff is not high, and the quality of life and psychological state of the patients are significantly lower than the normal population. In addition, most patients with uremia will have varying degrees of malnutrition before undergoing PD, mainly including hypoproteinemia, hyperphosphatemia, and anemia. After uremia patients receive PD treatment, although the degree of malnutrition is significantly improved compared with that before dialysis, the patients still suffer from malnutrition, which may increase the risk of cardiovascular events and death in the long-term [6]. Therefore, how to improve the therapeutic effect and nutritional status of uremia patients undergoing PD has become one of the hot issues in the medical field.

Mindfulness-based stress reduction (MBSR) was established by Dr. Jon Kabat-Zinn in 1979. MBSR is a systematic intervention method that takes mindfulness as the basis and relaxes individuals' body and mind through meditation and breathing training [7]. MBSR aims to focus on the individual, strengthen the emotional management, improve the physical and mental regulation ability of the individual, and uncritically devote them to and accept themselves, so as to achieve the purpose of alleviating the pain of the disease and reducing the inner pressure [8]. MBSR is intended to assist general medical behavior and has played an important role in the treatment of cancer, diabetes, mental illness, and other diseases [9–11]. Kral's team [12] found that MBSR plays a positive role in reshaping the brain network and improving memory function and bad mood. The results of the Reich team [13] proved that MBSR can improve the symptom clusters in breast cancer patients, including pain, psychology, fatigue, and cognition, and the beneficial effects of MBSR intervention can last for several weeks.

Solution-focused brief therapy (SFBT) is an intervention mode that focuses the problem on the positive aspects of the individual and guides the individual to solve the problem by exploring potential ability. It can enhance self-management ability and effectively reduce negative emotions, which has become a central issue in clinical research [14]. Gan's team [15] reported that SFBT has a good practical application effect in the family rehabilitation of adolescents with brain injury. SFBT can provide emotional support and is a promising psychological intervention. Wichowicz's team [16] found that the use of SFBT can reduce the intensity of depression and anxiety and improve self-efficacy in stroke patients, and it is simple, effective, and economical.

MBSR and SFBT play an important role in the management of many diseases at home and abroad. However, studies on the efficacy of MBSR combined with SFBT in patients with PD with uremia have not been reported. Therefore, the purpose of this study was to investigate the nursing effect of MBSR combined with SFBT in patients with uremia undergoing PD and to observe the changes of patients' nutritional status, so as to provide evidence for clinical application.

## 2. Materials and Methods

### 2.1. Research Object

A prospective study was conducted on 108 uremia patients undergoing PD who were admitted to the First People's Hospital of Wenling from March 2018 to December 2020. In accordance with the wishes of the patients, according to random number method, the patients were divided into control group (*n* = 54) and experimental group (*n* = 54).

#### 2.1.1. Inclusion Criteria

Inclusion criteria were as follows: adult patients; all of them meeting the diagnostic criteria for uremia [17] and treated with PD; dialysis time >3 months; giving informed consent to this study; clear consciousness; and basic understanding or reading and writing skills.

#### 2.1.2. Exclusion Criteria

Exclusion criteria were as follows: people with other critical illnesses; combination with mental illness; persons with communication disorders; patients who did not have the education level that could communicate normally; and people who cannot cooperate or withdraw from the research halfway.

### 2.2. Research Methods

#### 2.2.1. Control Group

Patients were given routine care. The nurses explained to the patients the relevant knowledge of uremia disease, the principle and precautions of peritoneal dialysis, the mechanism of action, and the use of therapeutic drugs; instructed patients to monitor their own diseases and improve their ability to take care of themselves; guided patients to face the disease and implemented psychological comfort; and instructed patients to supplement nutrition and exercise properly. The intervention was continued for 6 months, once a month.

#### 2.2.2. Experimental Group

Patients were given MBSR combined with SFBT. The MBSR and SFBT teams were established. The teams consisted of 6 medical staff, 4 nurses and 2 medical staff with the qualifications of the national grade II psychological counseling teacher. The team members were trained on MBSR and SFBT, so as to master the purpose, content, and precautions of the intervention and to take up the post after passing the assessment. A special relaxation room was established, the appropriate temperature and humidity were adjusted, and MBSR and SFBT intervention was carried out in a quiet and comfortable environment.

1. MBSR: Intervention with patients in a group manner. The intervention lasted for 6 months, 4 times a month, 30–45 min each time. ① Mindfulness training: In the quiet state of the ward, patients were instructed to take a comfortable sitting position, closed the eyes, and gradually relaxed the body from the feet to the head. The patients were instructed to focus their attention on breathing, adjusted breathing, maintained breathing regularity, listened to breathing sounds quietly, counted the number of breaths silently, and paid attention to the ups and downs of the abdomen. Through soothing language and music playing, patients were guided to relax and adjust their own psychology. ② Mindfulness meditation: The patients were instructed to practice mindfulness meditation and learn the basic core content of mindfulness training. During meditation, patients should bring mindfulness breathing and posture into the meditation and observe the thoughts and events emerging in their minds. Patients were instructed to feel the current emotions, thoughts, body, and other feelings, listen to their inner thoughts, and give psychological counseling and they were guided to eliminate distracting thoughts. Patients were instructed to imagine themselves in the most relaxing environment and were guided to observe the contents of meditation; the patients were made to accept the occurrence of disease and the current situation of receiving treatment, and the physical and mental state of the patients was improved.
2. SFBT: Intervene with the patient on a one-to-one basis. The intervention lasted for 6 months, once a month, 60 min each time. ① Described the problem: The staff communicated with the patient actively, gained the trust of the patient, and introduced the relevant knowledge of peritoneal dialysis to the patient in easy-to-understand language. They identified the specific problems that need to be solved, and the difficulties and the causes of the problems were understood. They found out in detail what the patient had done in the past to solve the problem and guided the patient to describe their personal feelings, including “what was your previous state like?” “how did you feel about receiving peritoneal dialysis?” “do you think peritoneal dialysis treatment is working for you?” ② Goal construction: The staff set up reasonable and feasible goals according to the patients' existing problems, timely explained the patients' disease progress, treatment projects, treatment costs, and so forth, encouraged the patients to self-regulate negative emotions, diverted the patients' attention to the disease itself, and helped the patients build up the confidence and courage to overcome difficulties. The medical staff and the patient discussed the problem together, such as “how would you be different now if the problem was resolved?” ③ Explored the exception: After the goal was constructed, they started to explore the exception, guided the patient to recall the problem that they had solved or accidentally solved, summarized the experience of solving similar problems, discussed the past successful experience with the patient, and analyzed how to make the past “exception” again, for example, “how did you do when the problem was not serious in the past?” ④ Gave feedback: They found out the advantages of the patients, supported the previous efforts made by patients, and gave them positive feedback such as praise and encouragement when patients achieved certain results in the process of achieving goals. Patients should be encouraged to continue to actively receive treatment. If the outcome of care was not obvious or the improvement of psychological status was not obvious, the medical staff should review the feasibility of setting goals and adjust them according to the actual situation. ⑤ Evaluated progress: They asked the patients if they were aware of their progress, for example, “how was your past state, then how is your current state?” They fully affirmed the progress made by the patient in the process of peritoneal dialysis treatment, guided the patients to reach the next goal, and helped patients summarize their experience. They built up confidence and moved further towards the desired goal.

### 2.3. Research Tools

Before and after the intervention, the researchers explained the purpose and content of the study to the patients, conducted the survey by filling out the questionnaire, and guided the patients to complete the questionnaire. The effective recovery rate of the questionnaire was 100%.

#### 2.3.1. Clinical Data

The clinical data such as age, gender, body mass index (BMI), dialysis time, and level of education were recorded.

#### 2.3.2. Biochemical Indicators

The fasting venous blood of the two groups was collected, and serum hemoglobin (Hb), serum albumin (ALB), and urea clearance index (*KT*/V) were detected: *KT*/*V*=−In(*R* − 0.008*∗T*+4 − 3.5*∗R*)*∗*UF/*W*; *K* is clearance rate, *T* is treatment time, *V* is urea distribution volume, *R* is urea nitrogen before dialysis/urea nitrogen after dialysis, UF is ultrafiltration rate, and *W* is dry weight.

#### 2.3.3. Complication

The occurrences of peritonitis, peritoneal hernia, abnormal peritoneal function, infection at the exit, and other complications were recorded in the two groups.

#### 2.3.4. Compliance

The compliance of the two groups was evaluated using the treatment compliance scale made by our hospital. There were 10 questions in the scale, including 4 dimensions of dialysis treatment, reasonable diet, emotional stability, and follow your doctor's prescription. Each item was scored between 0 and 25 points, and the full score was 100 points. The higher the score, the higher the individual's clinical compliance. The content validity index of our self-made questionnaire was 0.85, and the internal consensus reliability coefficient of Cronbach's *α* was 0.86, which has good reliability and validity.

#### 2.3.5. Nutritional Status

The malnutrition inflammation score (MIS) system was used to evaluate the nutritional status of the two groups. There were 10 questions in the system, with a total score of 0–30 points: 0 points, normal nutrition; 1–8 points, mild malnutrition; 9–18 points, moderate malnutrition; and >19 points, severe malnutrition. The higher the score, the worse the nutritional status of the individual. Cronbach's *α* coefficient of the scale was 0.785.

#### 2.3.6. Quality of Life

The Kidney Disease and Quality of Life-36 (KDQOL-36) questionnaire was used to evaluate the quality of life of the two groups. The questionnaire consists of 36 questions, including a general section and a specific section. The general part contains 12 questions, including physical health and psychological health. The specific section contained 24 questions, including three dimensions: kidney burden, symptoms and discomfort, and the effects of kidney disease. The total score ranged from 0 to 100 points. The higher the score, the better the quality of life. Cronbach's *α* coefficient of the scale was 0.792.

### 2.4. Statistical Methods

SPSS 22.0 software was used for analysis, measurement data were expressed as $\bar{x}\pm s$, and *t*-test was used for comparison. Count data was expressed as %, and *χ*^2^ test was used for comparison. *P* < 0.05 was statistically significant.

## 3. Results

### 3.1. Comparison of Clinical Data between the Two Groups

There were no significant differences in age, gender, BMI, dialysis time, and level of education between the two groups (*P* < 0.05), as illustrated in Table 1.

### 3.2. Comparison of Biochemical Indicators between the Two Groups

Compared with the situation before intervention, serum Hb level in the control group was increased after intervention, and serum Hb, ALB levels, and *KT*/*V* in the experimental group were increased after intervention. After intervention, the serum Hb, ALB levels, and *KT*/*V* of the experimental group were higher than those of the control group (*P* < 0.05), as illustrated in Figure 1.

### 3.3. Comparison of Complications between the Two Groups

Compared with the control group, the experimental group has a lower incidence of complications (*P* < 0.05), as illustrated in Figure 2.

### 3.4. Comparison of Compliance between the Two Groups

Compared with the situation before intervention, the compliance scores of the experimental group were increased after intervention. After intervention, the compliance score of the experimental group was higher than that of the control group (*P* < 0.05), as illustrated in Figure 3.

### 3.5. Comparison of Nutritional Status between the Two Groups

Compared with the situation before intervention, the MIS scores of the two groups were reduced after intervention. After intervention, the MIS scores of the experimental group were lower than those of the control group (*P* < 0.05), as illustrated in Figure 4.

### 3.6. Comparison of Quality of Life between the Two Groups

Compared with the situation before intervention, the KDQOL-36 scores of the two groups increased after intervention. After intervention, the KDQOL-36 scores of the experimental group were higher than those of the control group (*P* < 0.05), as illustrated in Figure 5.

## 4. Discussion

Uremia patients undergoing PD not only need to bear the physical trauma caused by the disease itself, such as insomnia, thirst, and physical pain, but also need to bear the economic burden caused by long-term PD treatment. As a result, patients are often accompanied by huge psychological and physical dual pressure, resulting in emotional disorders, reduced treatment compliance, and reduced living standards [18]. Therefore, it is important to find a scientific and effective intervention method to improve the nursing effect of uremia patients undergoing PD.

Hb is the main component of red blood cells, and it can bind with oxygen and transport oxygen and carbon dioxide, which can reflect the degree of anemia. ALB is synthesized by the liver and is the main protein component of normal human serum total protein. Serum Hb and ALB levels can be used as indicators to monitor the nutritional status of PD patients, and the judgment results are relatively objective, reliable, and easy to detect. *KT*/*V* can be used as an indicator to reflect the effectiveness of dialysis, and measuring *KT*/*V* has certain significance in determining whether PD treatment is adequate. In this study, after intervention, serum Hb, ALB levels, and *KT*/*V* of the experimental group were significantly increased, and the incidence of complications of the experimental group was lower than that of the control group. This indicated that MBSR combined with SFBT has a better nursing effect in uremia patients undergoing PD. MBSR is an intervention method for the human body to self-regulate psychological stress. This method awakens the body's attention and concentration based on the concept of Buddha-Zen thought, so that people can pay attention to the current situation, but does not make subjective comments on it. MBSR can guide the uremia patients undergoing PD to observe the contents of meditation, so that the patients can accept the occurrence of disease and the current situation of receiving treatment, which can enable the patient to fully understand their own disease and improve the degree of cooperation in treatment. At the same time, during the MBSR intervention process, the medical staff guide uremia patients to gradually relax their body from foot to head and feel the current emotions and thoughts, which can reduce the individual's psychological pressure, help them establish positive thoughts and emotions, correct the deviation of the patients' cognition and keep them in a good state of mind to continue treatment, and then realize the adjustment of physical and mental health [19]. SFBT is based on making full use of the resources of the uremia patients undergoing PD, focusing on the positive aspects of the patients, and building solutions together with the patients, as well as stimulating patients' subjective enthusiasm to solve their own problems, so that patients actively participate in disease management, and discovering the patients' own potential and resources to the greatest extent, so as to improve clinical symptoms. SFBT can unearth the potential of uremia patients undergoing PD, standardize health management methods, and guide patients to formulate scientific and feasible plans to correctly recognize and manage their own diseases, so that patients can face the diseases and life more positively and optimistically, and thus improve the treatment effect [20]. We combined MBSR and SFBT to apply them to the uremia patients undergoing PD; both models were based on patients. On the one hand, the staff guided patients to relax and eliminate distracting thoughts; on the other hand, they mobilized patients' resources and potential to make them actively participate in the decision-making of the nursing plan. This is conducive to guiding patients to actively participate in improving their own adaptability, improving renal anemia, improving nutritional status, reducing complications, and helping patients recover social function to the greatest extent.

In clinical practice, traditional nursing intervention models are usually implemented for patients with uremia undergoing PD. Although the traditional nursing intervention model has a certain nursing effect on patients, the nursing work of this method is one-sided, and the intervention method is not detailed enough, which leads to the traditional nursing method not meeting the requirements of patients. Our physicians performed breathing exercises, muscle relaxation, sitting quietly, meditation, focusing on problems, building goals, and giving feedback and other measures to the uremia patients undergoing PD. The results found that, after the intervention, the compliance score and KDQOL-36 score of the experimental group were higher than those of the control group. MBSR guides patients to relax their minds and bodies, eliminate distracting thoughts, accept themselves noncritically, and face the disease correctly with a peaceful and positive attitude, thereby reducing the interference of bad thoughts, enhancing the level of mindfulness, and improving patients' compliance. At the same time, SFBT can effectively correct the patient's bad mood, make the patient maintain good state of mind, strengthen the patient's treatment compliance and enthusiasm, enable the patient to actively cope with the problem, effectively reduce anxiety and depression, reduce the burden on the kidney, relieve symptoms and discomfort, and reduce the influence of the kidney disease for life, which in turn improves the quality of life.

Patients with uremia will lose a large number of nutrients from the peritoneal dialysis fluid when undergoing PD. If they cannot take nutrients absorbed scientifically and supplement the necessary substances in time, long-term PD treatment may cause adverse consequences such as malnutrition, hypokalemia, and low resistance, affecting the treatment effect of patients. Studies have shown that malnutrition is an independent risk factor affecting the prognosis of PD patients, and malnutrition patients have a higher mortality rate [21]. The MIS score is a scoring system developed on the basis of the dialysis malnutrition score, which can more accurately assess the severity of malnutrition in PD patients, and the efficiency of diagnosing the malnutrition in PD patients was 100% [22]. Our results suggested that MBSR combined with SFBT can improve the nutritional status of patients. For patients with uremia undergoing PD, the application of MBSR is beneficial to stimulate their inner strength, so that emotions can be positively controlled, reduce the patient's mental stress, and gradually restore their overall regulation ability to normal. MBSR enables patients to better feel their own physical changes and guides patients to face their disease with a calm mood and effectively control the emotional and physical discomfort, so as to prevent patients from suffering from anemia, malnutrition, and other unhealthy conditions. In addition, SFBT can make patients with uremia actively participate in their own management, causing patients to shift their attention to active treatment, and use a variety of methods to distract patients' attention, with the characteristics of subjectivity and enthusiasm, so as to achieve positive nursing goals. After the application of SFBT, medical staff introduce uremia knowledge in detail to patients with uremia, provide adequate health education, help them understand the importance of PD treatment, help them develop good behavior and lifestyle, and then reduce the risk factors affecting health and improve the nutritional status of the body.

## 5. Conclusion

MBSR combined with SFBT has a good nursing effect in uremia patients undergoing PD and can increase the patient's treatment compliance, improve the quality of life, and improve the nutritional status. The sample size of this study is small, and no comparative study was conducted on factors such as marriage, occupation, and average monthly income of the enrolled patients. The results obtained have certain limitations. We need to further improve and supplement the research methods in the future and consider the interference of other factors in the study.

## Figures and Tables

**Figure 1:** Comparison of biochemical indicators between the two groups. Note: compared with the situation before intervention, ^*∗*^*P* < 0.05; compared with the control group, ^#^*P* < 0.05.

**Figure 2:** Comparison of complications between the two groups. Note: compared with the control group, ^#^*P* < 0.05.

**Figure 3:** Comparison of compliance between the two groups. Note: compared with the situation before intervention, ^*∗*^*P* < 0.05; compared with the control group, ^#^*P* < 0.05.

**Figure 4:** Comparison of nutritional status between the two groups. Note: compared with the situation before intervention, ^*∗*^*P* < 0.05; compared with the control group, ^#^*P* < 0.05.

**Figure 5:** Comparison of quality of life between the two groups. Note: compared with the situation before intervention, ^*∗*^*P* < 0.05; compared with the control group, ^#^*P* < 0.05.

**Table 1:** Comparison of clinical data between the two groups (*n*, %).

Clinical data	Control group (*n* = 54)	Experimental group (*n* = 54)	*χ*^2^ value	*P* value
*Age (years)*				
20–45	20 (37.04%)	24 (44.44%)	0.614	0.433
46–70	34 (62.96%)	30 (55.56%)		
*Gender*				
Male	29 (53.70%)	27 (50.00%)	0.148	0.700
Female	25 (46.30%)	27 (50.00%)		
*BMI (kg/m*^*2*^)				
<24	28 (51.85%)	25 (46.30%)	0.333	0.564
≥24	26 (48.15%)	29 (53.70%)		
*Dialysis time (years)*				
1–3	17 (31.48%)	19 (35.19%)	0.687	0.709
4–6	19 (35.19%)	15 (27.78%)		
7–10	18 (33.33%)	20 (37.04%)		
*Level of education*				
Junior high school and below	18 (33.33%)	19 (35.19%)	0.381	0.827
High school	24 (44.44%)	21 (38.89%)		
Junior college and above	12 (22.22%)	14 (25.93%)		

## Data Availability

The data used to support the findings of the study are available from the corresponding author upon request.

## References

[1] Sheerin N. S., Glover E. (2019). Haemolytic uremic syndrome: diagnosis and management. *F1000Research*.

[2] Formeck C., Swiatecka-Urban A. (2019). Extra-renal manifestations of atypical hemolytic uremic syndrome. *Pediatric Nephrology*.

[3] Fülöp T., Zsom L., Tapolyai M. B. (2017). Peritoneal dialysis: the unique features by compartmental delivery of renal replacement therapy. *Medical Hypotheses*.

[4] Watanabe Y., Okada H. (2018). Effect of combined peritoneal dialysis and hemodialysis on health-related quality of life. *Contributions to Nephrology*.

[5] Cirillo L., Cutruzzulà R., Somma C. (2018). Depressive symptoms in dialysis: prevalence and relationship with uremia-related biochemical parameters. *Blood Purification*.

[6] Usta M., Ersoy A., Ayar Y., Budak F. (2020). The relationship between lymphocyte subsets, nutritional status and tuberculin reactivity in continuous ambulatory peritoneal dialysis and hemodialysis patients. *International Urology and Nephrology*.

[7] Botha E., Gwin T., Purpora C. (2015). The effectiveness of mindfulness based programs in reducing stress experienced by nurses in adult hospital settings: a systematic review of quantitative evidence protocol. *JBI Database of Systematic Reviews and Implementation Reports*.

[8] Greeson J. M., Zarrin H., Smoski M. J. (2018). Mindfulness meditation targets transdiagnostic symptoms implicated in stress-related disorders: understanding relationships between changes in mindfulness, sleep quality, and physical symptoms. *Evidence-based Complementary and Alternative Medicine: ECAM*.

[9] Cillessen L., Johannsen M., Speckens A. E. M., Zachariae R. (2019). Mindfulness‐based interventions for psychological and physical health outcomes in cancer patients and survivors: a systematic review and meta‐analysis of randomized controlled trials. *Psycho-Oncology*.

[10] Woods-Giscombe C. L., Gaylord S. A., Li Y. (2019). A mixed-methods, randomized clinical trial to examine feasibility of a mindfulness-based stress management and diabetes risk reduction intervention for african Americans with prediabetes. *Evidence-based Complementary and Alternative Medicine*.

[11] Bulzacka E., Lavault S., Pelissolo A., Bagnis Isnard C. (2018). Mindful neuropsychology: repenser la réhabilitation neuropsychologique à travers la pleine conscience. *L’Encéphale*.

[12] Kral T. R. A., Schuyler B. S., Mumford J. A., Rosenkranz M. A., Lutz A., Davidson R. J. (2018). Impact of short-and long-term mindfulness meditation training on amygdala reactivity to emotional stimuli. *NeuroImage*.

[13] Reich R. R., Lengacher C. A., Alinat C. B. (2017). Mindfulness-based stress reduction in post-treatment breast cancer patients: immediate and sustained effects across multiple symptom clusters. *Journal of Pain and Symptom Management*.

[14] Franklin C., Zhang A., Froerer A., Johnson S. (2017). Solution focused brief therapy: a systematic review and meta-summary of process research. *Journal of Marital and Family Therapy*.

[15] Gan C., Ballantyne M. (2016). Brain injury family intervention for adolescents: a solution-focused approach. *NeuroRehabilitation*.

[16] Wichowicz H. M., Puchalska L., Rybak-Korneluk A. M., Gąsecki D., Wiśniewska A. (2017). Application of solution-focused brief therapy (SFBT) in individuals after stroke. *Brain Injury*.

[17] Alseiari M., Meyer K. B., Wong J. B. (2016). Evidence underlying kdigo (kidney disease: improving global outcomes) guideline recommendations: a systematic review. *American Journal of Kidney Diseases*.

[18] Xia X., Wu X., Zhou X., Zang Z., Pu L., Li Z. (2021). Comparison of psychological distress and demand induced by COVID-19 during the lockdown period in patients undergoing peritoneal dialysis and hemodialysis: a cross-section study in a tertiary hospital. *Blood Purification*.

[19] Bennett P. N., Ngo T., Kalife C., Schiller B. (2018). Improving wellbeing in patients undergoing dialysis: can meditation help?. *Seminars in Dialysis*.

[20] Beyebach M., Neipp M. D. C., García-Moreno M., González-Sánchez I. (2018). IMPACT of nurses′ solution-focused communication on the fluid adherence of adult patients on haemodialysis. *Journal of Advanced Nursing*.

[21] Maraj M., Kuśnierz-Cabala B., Dumnicka P. (2018). Malnutrition, inflammation, atherosclerosis syndrome (MIA) and diet recommendations among end-stage renal disease patients treated with maintenance hemodialysis. *Nutrients*.

[22] Brandão da Cunha Bandeira S., Cansanção K., Pereira de Paula T., Peres W. A. F. (2020). Evaluation of the prognostic significance of the malnutrition inflammation score in hemodialysis patients. *Clinical Nutrition ESPEN*.

